# Correlation of TET-2 Levels with Disease Evaluation in AMI Patients

**DOI:** 10.1155/2022/9983071

**Published:** 2022-07-31

**Authors:** Qinglei Wang, Shan Fu, Shucheng Li, Xiansheng Huang, Hong Wang

**Affiliations:** Department of Cardiology, Affiliated Hospital of Chengde Medical University, Chengde 067000, Hebei, China

## Abstract

**Objective:**

To investigate the expression levels of Ten-Eleven Translocation-2 (TET-2) in patients with acute myocardial infarction (AMI) and correlations of TET-2 levels with disease severity.

**Methods:**

A total of 150 patients with confirmed AMI were included in this study. According to the number of coronary artery lesions, the patients were divided into a single lesion group, two lesion group, and three lesion group. According to the Gensini scores, these patients were also assigned into three groups: the low-risk group, middle-risk group, and high-risk group. 150 patients without AMI confirmed by coronary angiography were included in the control group in the same period. TET-2 and cardiac troponin T (cTNT) levels were detected by ELISA analysis and compared among different groups. Pearson's correlation analysis was used to evaluate the correlations of TET-2 levels and cTNT levels/Gensini scores. The levels of TET-2 in AMI patients increased remarkably with the increase of disease severity. Patients in the single lesion group or low-risk group had the lowest levels of TET-2. Pearson correlation analysis indicated that TET-2 levels were positively associated with cTNT levels and Gensini scores, respectively (all *P* < 0.001).

**Conclusion:**

The levels of TET-2 were upregulated in AMI patients and positively correlated with cTNT levels or Gensini scores, suggesting that the examination of TET-2 expression levels could be exploited for predicting the disease severity.

## 1. Introduction

Acute myocardial infarction (AMI) is a common cardiovascular disease, which is considered as one of the leading reasons for mortality and morbidity worldwide [1]. It was reported that the incidence rate of AMI was increased year by year with the aging population, life pace acceleration, and lifestyle change [2]. It was estimated that the mortality rate of cardiovascular disease ranked third in human death [3, 4]. The etiology and pathogenesis for AMI are very complex. It is mainly caused by an acute interruption of myocardial blood. In clinical practices, coronary angiography plays a critical role in evaluation of disease severity for AMI. The evaluation of the disease severity for these patients would help in guiding clinical treatment and assessing prognosis. Cardiac troponin T(cTNT) is generally involved in myocardial necrosis and has become a gold standard biomarker for AMI. However, the increased levels of cTNT may be caused by the following diseases such as myocarditis, renal failure, chest trauma, heart failure, and so on [5]. Therefore, there is an urgent requirement for new biomarkers in the early stages of AMI to reduce the period of diagnosis and improve the prognosis in these AMI patients.

In recent years, as in-depth studies on coronary heart diseases show, DNA 5-methylcytosine levels have been closely associated with the development and progression of atherosclerosis [6, 7]. It was reported that enzymatic pathways involved in DNA methylation and the important role of ten-eleven translocation (TET) proteins in DNA methylation were confirmed [8]. TET family members consisted of TET-1, TET-2, and TET-3. Many studies showed that the presence of TET proteins had been confirmed in tissues in which the DNA demethylation process occurred. In addition, among these members, TET-2 was positively correlated with the phenotypic transformation of vascular smooth muscle cells [9]. Liu et al. reported that the reduction of TET-2 levels was found in human atherosclerosis tissues [10]. Fuster et al. also revealed that TET-2 mutation in somatic cells could significantly boost the development of atherosclerosis in mice [11]. However, it is unknown about the relationship between the expression changes of TET-2 and the disease severity in patients with AMI.

In this study, the serum levels of TET-2 were detected in patients with AMI, and its relationship with disease severity was evaluated. This study would bring some insights into effective biomarkers for evaluating disease severity and predicting prognosis in AMI patients.

## 2. Materials and Methods

### 2.1. Subjects

A total of 150 AMI patients admitted to our hospital from July 2020 to September 2021 were selected as the research subjects included in this study. The inclusion criteria were as follows: the age was over 18 years old. Patients met the diagnostic criteria of myocardial infarction, which was confirmed by the coronary angiograms; patients underwent the examination of coronary angiograms and serum cTNT levels [12], and the severity of AMI was graded as follows: single lesion, two lesions, and three lesions. According to the Gensini scores [13], disease severity grading for AMI patients was as follows: the low-risk group, middle-risk group, and high-risk group. All the patients signed informed consent forms, and this study was approved by the Ethics Committee of our hospital.

The relationship between the coronary artery Gensini score and the left ventricular function was analyzed. The relationship between the Gensini score and the left ventricular function was analyzed. The coronary artery Gensini score was 0–165, with an average of (22.6 ± 4.7). With the increase of the coronary artery Gensini score, LVEF gradually decreased, LVEDV and LVESV gradually increased, and the difference between the groups was statistically significant (P0.01).

### 2.2. Detection of Serum cTNT and TET-2 Levels

The serum levels of cTNT and *TET-2* in patients were compared among different groups. At 12 h after fasting, 2 mL venous blood in each patient was drawn from the elbow vein in the morning and kept in the ethylene diamine tetraacetic acid (EDTA) anticoagulant tube. The plasma was separated by centrifuging at 3500 r/min for 10 min and then stored at −20°C. The levels of cTNT and TET-2 were examined by the ELISA method, strictly following the instructions on ELISA kits (R&D Systems, USA).

ELISA is the most reliable kit on the market and the most cited kit in the published literature. It has 700 target analytes and covers 12 species. Following our high quality production and performance standards, our ELISA products can achieve the desired results every time. Quantikine ELISA is a ready to use kit. The DuoSet development kit provides users with greater flexibility.

- High quality results with limited budget and maximum ELISA selection range
- IC (intracellular) ELISA development system
- Detection of intracellular molecules in cell lysates by Sandwich ELISA
- IC (intracellular) phosphorylation ELISA development system
- Detection of phosphorylated molecules in cell lysates by Sandwich ELISA
- ELISA/test AIDS
- Microplate, cleaning solution, diluent, test reagent, termination solution, sample collection kit, and other products
- View all DuoSet development systems
- Search in the largest kit menu to create your own ELISA test.

### 2.3. The Results of Coronary Angiography Evaluated by Gensini Scores

Gensini scores were used to assess the results from coronary angiography of each patient. The scores were calculated based on different lesions: 5 points for the left main, 2.5 points for the proximal left anterior descending artery or circumflex artery, 1.5 points for the middle part of the left anterior descending branch, and 1.0 points for the distal left anterior descending branch, circumflex artery, and the right coronary artery, and the small branch is 0.5 points. The scores were also obtained according to the degree of stenosis in each coronary artery: 1%–25% coronary artery stenosis was 1 point, 26%–50% coronary artery stenosis was 2 points, 51%–75% coronary artery stenosis was 4 points, 76%–90% coronary artery stenosis was 8 points, 91%–99% coronary artery stenosis was 16 points, and complete occlusion in the coronary artery was 32 points. The scores for each lesion were calculated through coronary narrow degree integral multiplied by the lesion location scores. Gensini scores for each patient were the total amount of the scores from coronary artery lesions.

### 2.4. Statistical Analysis

Data analysis was conducted with SPSS software, version 23.0. The quantitative data were presented as the mean ± standard deviation (SD). One-way analysis of variance (ANOVA) was exploited for comparisons among three groups, while Student's *T* test was exploited for comparison between the two groups. The correlation analysis between TET-2 levels and cTNT levels/Gensini scores was performed by Pearson correlation analysis. The count data were expressed as percentages or cases, and the Chi-square test was exploited for comparison between the two groups. The logistic regression method was used to evaluate whether TET-2 was a risk factor for disease severity in AMI patients. *P* < 0.05 was considered a statistically significant difference.

## 3. Results

### 3.1. Comparison of General Data

There was no significant difference between the two groups for baseline data including age, sex, body mass index (BMI), hypertension, diabetes, hyperlipidemia, and smoke (*P* > 0.05), so the two groups are comparable, as shown in Table 1.

### 3.2. Comparison of cTNT and TET-2 Levels between the AMI Group and the Control Group

As shown in Table 2, the serum cTNT level in the control group was 78.4 ± 6.5 ng/L, while it was 3562.8 ± 429.1 ng/L in the AMI group. The serum cTNT level in the AMI group was obviously more than that in the control group, and there were significant differences between the two groups (*P* < 0.04). In addition, the serum TET-2 level in the AMI group was 10.4 ± 0.8 ng/mL, which was significantly higher than that in the control group (3.7 ± 0.5 ng/mL). There were statistical differences between the two groups (*P* < 0.05).

### 3.3. Serum Levels of TET-2

As seen in Figure 1, the serum levels of TET-2 in the single lesion group, two lesion group, and three lesion group were 4.8 ± 0.9 ng/mL, 8.9 ± 1.1 ng/mL, and 12.4 ± 1.2 ng/mL, respectively. Compared with the single lesion group, the serum levels of TET-2 in the two lesion group and three lesion group were significantly higher, and there were statistical differences (all *P* < 0.05). The serum levels of TET-2 in the three lesion group were remarkably higher than those in the two lesion group (*P* < 0.05). Moreover, the serum levels of TET-2 in the low-risk group, middle-risk group, and high-risk group were 3.9 ± 0.7 ng/mL, 9.4 ± 1.0 ng/mL, and 13.6 ± 1.2 ng/mL, respectively. Compared with the low-risk group, the serum levels of TET-2 in the middle-risk group and high-risk group were obviously higher, and there were significant differences (all *P* < 0.05). The serum levels of TET-2 in the high-risk group were obviously higher than those in the middle-risk group (*P* < 0.05).

### 3.4. Logistic Regression Analysis

The results of logistic regression analysis for severity grading of coronary artery lesions revealed that the values of OR for TET-2 were 1.702 (95%CI: 1.432–2.738). The serum TET-2 level was the independent risk factor for patients with AMI, and there were significantly statistical differences (*P* < 0.05), as shown in Table 3.

### 3.5. Correlation between TET-2 Levels and cTNT Levels/Gensini Scores

As shown in Figure 2, the correlation coefficient between TET-2 levels and *cTNT levels* was 0.746, and the significant differences were observed (*P* < 0.001). In addition, the statistically significant correlation was obtained between TET-2 levels and Gensini scores (*r*= 0.773, *P* < 0.001).

## 4. Discussion

AMI not only seriously threatens the life quality and physical and psychological health of patients but also exerts a significantly financial burden on the health care system. AMI is a condition which could be due to coronary artery disease or ischemic heart disease in conjunction. It occurs when the coronary artery is partially or totally occluded by the atherosclerotic plate ruptures and the developing thrombus, resulting in blood having no access to the heart [14, 15]. It was firstly proposed by Newman et al. in 1999 that atherosclerosis was associated with DNA methylation [16]. Many studies confirmed that abnormal DNA methylation was one of the main causes for the development of atherosclerosis [17]. DNA methylation could turn off the activity of certain genes, resulting in gene silencing. Some studies showed that decreased levels of genomic DNA methylation had been observed in human atherosclerotic plaques, atherosclerotic plaques from ApoE knockout mice, arterial neointima in New Zealand rabbit, and atherosclerotic tissues from the rabbit aortic arch [18]. Other studies reported that hypermethylation conditions were found in the whole genome of pathological tissue and peripheral blood cells from patients with coronary heart disease [19]. Moreover, the level of DNA methylation in the peripheral blood of patients with coronary heart disease was significantly increased [20]. DNA methylation plays an important role in the development of atherosclerosis.

To monitor the DNA methylation levels in AMI patients, this study focused the expression level of TET-2. TET proteins have been demonstrated to have appeared in the DNA demethylation process. TET-2 was reported to convert 5-methyl-cytosine to 5-hydroxymethyl-cytosine during DNA demethylation [21]. TET-2 mutations could result in the reduction of TET-2 enzymatic activity, which is correlated with changes in methylation profiles and epigenetic dysregulation [22]. The research studies regarding the role of TET-2 mostly focus on tumors. It was reported that TET-2 could regulate the global hydroxymethylation status and further participate in tumor progression in prostate cancer [23]. The downregulation of TET-2 was observed in hematologic malignancies. Zhang et al. demonstrated that TET-2 expression could act as a potential biomarker monitoring disease surveillance of patients with acute myeloid leukemia [24]. Among TET family members, TET-2 was the most highly expressed type in human coronary artery smooth muscle cells [25]. Under the stimulation of injury, the TET-2 level was significantly decreased in vascular smooth muscle cells. In addition, some studies showed that TET-2 was an important negative transcriptional suppressor of proinflammatory responses, and TET-2 function was associated with atherosclerosis development in mice through enhanced inflammatory responses [26]. Other studies demonstrated that there was a significant association between aging and TET-2 mutations [27, 28]. The present study showed that the serum levels of TET-2 were obviously upregulated in AMI patients and positively associated with disease severity of AMI, indicating that TET-2 could predict the disease severity of AMI and guide the clinical treatment.

In conclusion, this study suggested that the serum levels of TET-2 are significantly increased in patients with AMI and are associated with disease severity of AMI. However, the specific molecular mechanism of TET-2 in the pathogenesis of atherosclerosis remains unclear, requiring further experimental confirmation. Along with the deepening of research on DNA methylation, it would provide new directions for the treatment of coronary heart disease. [29].

## Figures and Tables

**Figure 1:** Comparison of serum levels of TET-2 among different groups. (a) Different lesion groups, compared with a single lesion,  ^*∗*^*P* < 0.05 and compared with two lesions, ^#^*P* < 0.05; (b) different risk groups, compared with the low-risk group,  ^*∗*^*P* < 0.05 and compared with the middle-risk group, ^#^*P* < 0.05.

**Figure 2:** The correlation analysis between TET-2 and cTNT/Gensini scores. (a) TET-2 levels were positively associated with cTNT levels. (b) TET-2 levels were positively associated with Gensini scores.

**Table 1:** The basic information of patients with ulcerative colitis.

Indexes	Control group (*n* = 150)	AMI group (*n* = 150)
Age (years)	66.4 ± 7.5	67.2 ± 8.1
Gender (male/female)	77/73	80/70
BMI (kg/m^2^)	21.1 ± 0.6	20.9 ± 0.4
Hypertension (n)	65	70
Diabetes (n)	25	34
Hyperlipidemia (n)	15	20
Smoke (n)	38	46

*Note.* AMI: acute myocardial infarction; BMI: body mass index.

**Table 2:** Comparison of serum levels of cTNT and TET-2 between the AMI group and the control group.

Groups	Cases (n)	cTNT (ng/L)	TET-2 (ng/mL)
Control group	150	78.4 ± 6.5	3.7 ± 0.5
AMI group	150	3562.8 ± 429.1 ^*∗*^	10.4 ± 0.8 ^*∗*^

*Note.* AMI: acute myocardial infarction; cTNT: cardiac troponin T; TET-2: Ten-Eleven Translocation-2; compared with the control group,  ^*∗*^*P* < 0.05.

**Table 3:** Logistic regression analysis for severity grading of coronary artery lesions in patients with AMI.

Factors	*β*	SE	Wald	*P*	OR	95%CI
TET-2	1.046	3.084	1.305	0.002	1.702	1.432–2.738

*Note.* TET-2: Ten-Eleven Translocation-2; SE: standard error; OR: odds ration; CI: confidence interval.

## Data Availability

The experimental data used to support the findings of this study are available from the corresponding author upon request.
